This article has been retracted.

# Economic affordability of food as a component of the economic security of Ukraine

**DOI:** 10.1371/journal.pone.0263358

**Published:** 2022-03-03

**Authors:** Tetiana L. Mostenska, Tetiana G. Mostenska, Eduard Yurii, Zoltán Lakner, László Vasa

**Affiliations:** 1 Faculty of Transport, Management and Logistics, National Aviation University, Kyiv, Ukraine; 2 Doctoral Studies in Economics and Business, Zaporizhzhia National University, Zaporizhzhia, Ukraine; 3 Department of Public, Corporate Finance and Financial Intermediation, Yurii Fedkovych Chernivtsi National University, Chernivtsi, Ukraine; 4 Doctoral School éf Economics and Regional Sciences, Hungarian University of Agriculture and Life Sciences, Gödöllő, Hungary; 5 Széchenyi István University, Győr, Hungary; Hungarian University of Agriculture and Life Sciences (MATE), HUNGARY

## Abstract

Economic security can be considered as an economic aspect of the life of an individual or household that provides the opportunity to achieve financial stability and improve living standards. In this context, understanding the impact of economic affordability of food on the economic security of the country is of great importance. The authors propose to use the indicator of economic affordability of food for in-depth analysis of the economic security of the country. Indicators that determine the level of economic affordability of food products in Ukraine for 2000–2018 are calculated. The regression analysis made it possible to establish a close relationship between the indicators of food expenditures and the level of GDP per capita, between the level of income and expenditure of food of decile groups. Correlation coefficients between the consumption of six basic foodstuffs and the level of per capita income in Ukraine are determined. The obtained indicators, which determine the economic affordability of food, allow us to conclude that there is a lack of economic protection at the level of individual low-income households. Overcoming economic instability and minimizing the possible consequences of the low level of economic affordability of food should become one of the main tasks of Ukraine’s economic security.

## 1. Introduction

In determining the state of economic security, a special place is given to its social component of ensuring the basic human right of accessing food in terms of the economic affordability of food. The authors propose to use the indicator of economic affordability of food for in-depth analysis of the state of economic security. This indicator most fully characterises the living standards of both the household and the individual through the ability to meet the energy needs of man; the ability to consume sufficient food; to meet the needs of the body in macro-and micro-nutrients, vitamins and minerals. The economic affordability of food affects the cost of food, consumption patterns as well as the quality of food. It also decisively affects the duration and quality of life.

The affordability of food determines the living standards of the population and affects the level of economic security. The task of the state is to help ensure that the income of the population is at a level sufficient enough to provide a buffer stock that will allow households to remain at a level above economic instability in case of adverse events, and also to form economic conditions that ensure the sufficiency of food consumption.

The purpose of the study was to determine the state of economic affordability of food as a component of economic security of Ukraine. Food affordability is one of the main components of food security. It determines the level of food consumption, balanced nutrition, quality and life expectancy.

To analyze the economic affordability of food, the authors studied the trends in food security in Ukraine as a whole and the indicator of economic affordability as a component of the Global Food Security Index. This approach allows, according to the authors, to understand better the existing problems in the country on the availability of food in households with different income levels, reduce social tension in society, create preconditions for economic security, identify factors that could potentially threaten economic security.

The authors proposed a system of indicators that allows to determine the economic affordability of food for Ukrainian households on the basis of official statistics of Ukraine and international organizations.

The study on the relationship between the level of consumption of certain foods and the level of income allows to calculate the required level of income, which will ensure the consumption of food at the level of rational norms and balance the food basket of Ukrainians.

## 2. Literature review

The state of economic security is a subject of special concern for statesmen and international organisations alike. This problem is studied by both individual scientists and research institutions. Economic security in publications is considered by scientists to be an economic category from two positions:

1. as a component of national security, which characterises the economic condition of the country and the ability to resist the negative impact of objective and subjective factors to achieve the macroeconomic goals of the country.
2. as an economic aspect of the life of an individual or household, which provides the ability to achieve financial stability and improve living standards.

Different approaches define different research objects. In the first approach, they are the economic system of the country; certain areas of state regulation—social, legal and political; and society (institutions, organisations, business entities, and population).

The first approach is typical for scientists from Ukraine and post-Soviet countries. With such an approach devoted scientific publications to the economic security definition, identification and characterisation of the destabilising effects of factors that threaten the sustainable development of the country. Researchers study the ability to guarantee the protection of national interests, the socially oriented development of the country as a whole; ensuring sufficient defense potential even under the most unfavorable conditions for the development of internal and external processes; ensuring the most efficient use of resources to neutralise threats and ensuring stability in contemporary conditions and in the future [1–13].

Within the second approach, the object of study includes the population, individuals, households, income and expenditure structure. This approach is typical for scientists representing scientific schools in European countries and the United States. However, despite the different approaches of scholars to the definition of economic security, it is considered part of the national interests of any country.

The characteristics of economic security from the standpoint of the second approach are considered in the following publications [14–24].

The article considers economic security from the standpoint of ensuring the welfare of the population at the level of individuals and households. With this approach, economic security can be defined as a complex socioeconomic category. The Business Dictionary defines economic security as “A situation of having a stable source of financial income that allows for the on-going maintenance of one’s standard of living currently and in the near future.” [25].

Yale University (USA) uses surveys to characterise the level of economic security in the context of determining the economic security of households and determining the Economic Security Index (ESI). The Economic Security Index (ESI) is “an integrated measure of insecurity that captures the prevalence of large economic losses among households” [19]. That is, the Economic Security Index (ESI) is an integrated indicator of insecurity, which shows how large is the total economic loss of the US population.

A more detailed approach to defining economic security is demonstrated by The International Committee of the Red Cross (ICRC). The ICRC defines economic security “as the ability of individuals, households or communities to cover their essential needs sustainably and with dignity. This can vary according to an individual’s physical needs, the environment and prevailing cultural standards. Food, basic shelter, clothing and hygiene qualify as essential needs, as does the related expenditure; the essential assets needed to earn a living, and the costs associated with health care and education also qualify” [26].

Scientists also devoted their studies to the issue of the economic security of the country through the level of economic security of households. They consider economic security from different points of view.

Berloffa and Modena [15] examine the impact of unemployment on household economic risk. This takes into account the composition of the household, income per household member, the expected damage associated with unemployment, and the dependency ratio of the inactive unemployed (IUDR), which determines the average number of people who are not included in the labor force.

The works of Beeferman [14], Goldstein [19], Morrone et al [22], Nissanov [27], Wheary, Shapiro, & Draut [28] are devoted to identifying areas for increasing the economic security of households by increasing income and identifying possible sources of such growth as state social policy.

Threats to economic security are investigated via the impact of income inequality on social well-being [29] particularly, due to compensation policy in business processes [30] development of the agriculture sector in the context of ensuring food security [21, 31–35] shadow economy influence on social safety [36] and shifts in inequality due to the impact of globalisation [37, 38].

The dependence of economic security not only on the availability of sufficient income to provide for life, but also on the access to necessary services such as utilities, transport, education, health care, housing, etc. is discussed in Gordon [39].

The analysis of scientific publications allowed us to draw conclusions about the correctness of the study of economic affordability of food products as a component of economic security of the country.

In the study of economic security, there are no common approaches to determining its state. The versatility of this concept implies the possibility of using a variety of evaluation methods. These methods can be based on quantitative or qualitative assessments. The state of economic security can be determined by single indicators; groups of indicators based on retrospective analysis; integrated indicators; and groups (systems) of indicators.

In the approach to assessing the level of economic security, Carroll & Samwick [40] built on the method of scenarios, which is based on the determination of possible combinations of states, of economic security and financial consequences arising under the influence of both positive and negative factors. The proposed scenarios take into account changes in the labour market and possible changes in the level of income and expenses.

One approach in which economic security can be based on is in determining the level of minimum basic consumption which is provided by basic income. In this case, economic security is considered at a level that should provide households with a standard of living that will not pose a threat to their economic security. At the same time, the approach to assessment is carried out through the structure of consumption for individual groups of households and the possibility of influencing the change of this structure [21].

In addition, assessments can be made on the basis of both macroeconomic (national population) and microeconomic indicators (individual or household level) [41].

Research by Carroll & Samwick is built on the study of household income dynamics. The authors use a standard life cycle model and a model of saving "buffer stock" [40].

Expert methods of assessing economic security are widespread. To determine economic security, Osberg & Sharpe [23, 41] uses household level data; indices of the economic insecurities produced by the hazards identified in Clause 25 of the UN Universal Declaration of Human Rights (i.e. unemployment, illness, widowhood, disability and old age); and the aggregation of these indices to an over-all measure of economic insecurity. “Economic insecurity is a term used to describe the uncertainty surrounding economic aspects of people’s lives. Clearly, this is a multi-faceted issue and a comprehensive formal definition that subsumes all possible aspects of it” [13, 42].

The issues of risks arising from declining incomes in different decile groups of households and their affecting of the state of their economic security are considered in the works of Dynan, Douglas, & Sichel [43].

The issue “how differences in personal income and food prices might jointly influence dietary intakes of key foods among men and women of diverse ages across both rich and poor countries” was studied in [44, p.9]. The female eating behavior and eating styles over different sociodemographic traits was also studied widely [45, 46].

The need to ensure the affordability of food in the definition of public policy was emphasized in the 5th Scottish Government’s Food Forum. The materials of the forum state “There is a need for food security to be given an increased emphasis in government policy. Food should be a specific focus for future policy” [47, p.96.].

However, despite the use of different methods of determining economic security, the level of households is characterised as the most important. Since the list of factors influencing the economic instability of households does not have an unambiguous definition, there is no single method for assessing economic security at the household level. There is an evolution of views on both the components and characteristics of economic security, and, accordingly, the methods of its evaluation [23, 48–50].

The publications of Ukrainian scholars do not consider the issue of economic security of the country from the standpoint of economic well-being of households, which negatively affects the formation of social policy of the country and the creation of preconditions for achieving economic security. Determining the state of economic security at the household level allows to characterize the existing problems, to identify factors that could potentially threaten the economic security of households.

## 3. Materials and methods

One of the indicators that determines the economic security of the country is the indicator of food security. At the same time, one of the key roles in the system of food security indicators of Ukraine is played by the indicator of food affordability.

The research was conducted in the context of studying the affordability of food at the level of households and individuals.

### 3.1. Quantitative indicators for statistical analysis

For the statistical analysis, the data of the State Statistics Service were used, collected as a result of the survey of living conditions of households, which were carried out on a separate network of respondents (private households) for the period 2015–2020 [51–55]. The volume of the annual sample of households for the survey of living conditions in 2015–2018 was 13,029 households. Starting from 2018, the number of households living in the temporarily occupied territory of the Autonomous Republic of Crimea, in the city of Sevastopol and part of the temporarily occupied territories of Donetsk and Luhansk oblasts is excluded from the survey. During this period, the sample is 12,228 households (Expenditure and Resources of Households of Ukraine). The analysis of the data allowed to determine the dynamics of indicators of economic affordability and the level of consumption of basic food products for the population of Ukraine in the study period.

In addition, to analyze macroeconomic indicators, data from the State Statistics Service of Ukraine for 2000–2020 were used [56–62], which made it possible to determine the relationship between the level of consumption of basic food products and the income of the population of Ukraine, to build a regression equation.

### 3.2. Methods

For the study, the authors studied approaches to assessing the economic affordability of food products.

Affordability allows you to find out information about the availability of food for the population. Economic affordability can be determined by a system of indicators that includes food consumption as a share of household expenditures, the share of the population living below the global poverty line, gross domestic product per capita, import tariffs on agricultural products, the availability of food security programs in the country, availability of funding for farming development programs and others. This approach to assessing the economic affordability of food is proposed when calculating the Global Food Security Index [63].

Dorward, A. proposes to assess the economic affordability of food through changes in real incomes as a result of changes in food prices for the most vulnerable groups: the indicator of real food prices relative to real incomes [64].

The food affordability indicator is defined as one of the 17 food security indicators in [65] and is calculated through three indicators that can be defined at different levels: (country, region, household, individual):

Quantity—the adequacy of food, which is determined by the caloric content of food;
Quality—is determined by the quality of food (diversity, adequacy, sufficiency, overall balance);
Stability—is determined by the stability of availability, access and consumption, including the relationship with price changes.

There is an approach to determining the economic affordability of food through the ratio of real wages and food prices [66]. The definition of economic affordability indicators is also considered in the works [67, 28].

The study of economic security assessment methods presented in [17, 21, 23, 40–43, 48] allowed the authors to use a set of quantitative (dynamic and comparative analysis, regression analysis, comparisons, structural analysis) when studying the issue of economic affordability of food at the household level as a component of economic security and qualitative evaluation methods (household survey results). The study is based on the definition of a system of indicators of economic affordability of food, which characterizes the current state of economic affordability of food in Ukrainian households on the basis of official statistics of Ukraine and international organizations.

The authors of the article propose to consider economic affordability through a system of indicators, including GDP per capita; Expenses / incomes per household per year; Costs / incomes per person per year, Food costs’; Food costs per person per year. Indicators for comparative analysis were calculated in two currencies, hryvnias and US dollars.

To characterize the changes and forecast the state of consumption of certain foods, the authors determined the equation of the relationship between the consumption of certain foods and the income level of the population.

## 4. Results

Social stability is one of the most important assessments of the country’s economic security. Social policy, which forms social stability in the country, must ensure the economic security of individuals and households. One of the biggest threats in this context is the significant income differentiation of different population groups. The value of the decile coefficient as the ratio of 10% of the richest and 10% of the poorest citizens of the country demonstrates the differentiation of the population by the level of per capita income. If this ratio exceeds ten fold, then society enters a zone of social tension. [68].

Indicators characterising the distribution of households by the level of per capita equivalent total income are presented in Table 1.

**Table 1:** Indicators characterizing the distribution of households by income level.

Indicators	2015	2016	2017	2018	2019	2020
Concentration factor (Ginny index)	0.243	0.244	0.232	0.238	0.265	0.260
Decile coefficient of differentiation of total incomes, times	2.8	2.8	2.6	2.9	3.3	3.1
The ratio of total income of the most and least well-off 10% of the population (decile ratio of funds), times	5.0	4.9	4.5	4.7	4.9	4.9

Source: calculated by the authors. Source: [55, 58–61].

According to official statistics, the almost five-fold gap between the incomes of the richest and poorest citizens of Ukraine is not evidence of an economic threat. However, in 2020, there were almost 29,2% of citizens in Ukraine with average per capita equivalent total incomes below the actual subsistence level. Against this background, the number of Ukrainians who declared an income exceeding one million hryvnias is growing from 1,061 citizens in 2017 to 4,817 in 2018. The indicator for 2020 is 3,150 people. Further stratification of the population in terms of income may become a threat to economic security at the household level.

Based on the above, in order to ensure economic security, the political and institutional decisions of the government should be aimed at ensuring social justice and improving the conditions of the most vulnerable segments of the population.

One of the components of the country’s economic security is food security. Food security is seen as the ability of individuals, households, and communities to acquire food that is sufficient, reliable, nutritious, safe, acceptable, and sustainable [65, 69–72]. Considering this, the issue of food availability is important from the point of view of ensuring economic security. Food affordability is one of the main indicators that characterises food security both at the national level and at the level of individual households and individuals. One of the indicators that determines the economic affordability of food is the level of income of the population.

Food access refers to the extent to which individuals are physically and economically able to obtain nutritious foods [3] and represents the consumer determinant of food security. Food access is determined by physical resources (including transport, time, and mobility, and the presence/absence/proximity of food-related facilities), financial resources, social support, and the skills and knowledge to make appropriate choices.

Scientific papers consider the two concepts of food affordability:

1. the ability to pay for healthy nutritious food.
2. food awareness—the knowledge and skills needed for food preparation and cooking.

This article examines the problem of affordability of food as a component of economic security through the ability to pay for healthy nutritious food. The rationale for this approach lies in the plane of the existing level of purchasing power of the population. The average monthly size of the legally established subsistence level in 2017 was UAH 1,603.67 and in 2020 –UAH 2,078.42 per person per month; the average monthly size of the actual subsistence level in 2017 was UAH 2,941.46 and in 2020 –UAH 3,847.21 per person per month. According to statistics, the number of poor people in Ukraine remains quite high. Households with per capita equivalent total income per month below the actual subsistence level in 2020 accounted for 29.5% of the total. At the same time, for households living in rural areas this indicator was at the level of 44.4% (Table 2).

**Table 2:** Distribution of households with per capita equivalent money income for a month below subsistence line, %.

	Share of households with per capita equivalent cash income per month is lower											
	the statutory established minimum subsistence level*						the actual subsistence minimum**					
	2015	2016	2017	2018	2019	2020	2015	2016	2017	2018	2019	2020
All households	9.4	9.3	6.4	4.1	2.6	3.0	60.7	63.1	48.0	38.8	30.8	29.5
including those living in:												
urban settlements	7.7	7.9	4.9	3.2	1.2	1.8	55.8	59.0	43.5	34.0	24,7	24,3
rural areas	13.0	12.2	9.3	6.1	5.2	4.8	70.6	71.6	57.2	48.7	45.4	44.4
Established minimum, hryvnia	1,227.3	1,388.1	1,603.7	1,744.8	1,902.1	2,078.4	2,257.0	2,642.4	2,941.5	3,262.7	3,660.9	3,847.2

Source: calculated by the authors. Source: [54, 58–60].

* Subsistence level is a value sufficient to ensure the normal functioning of the human body, maintaining its health set of foods, as well as a minimum set of non-food items and a minimum set of services necessary to meet basic social and cultural needs of the individual in accordance with the Law of Ukraine "On cost of living".

** Actual subsistence level—calculated monthly by the Ministry of Social Policy of Ukraine to monitor the dynamics of living standards in Ukraine on the basis of statistical data on the level of consumer prices.

A significant gap between the subsistence level and the actual subsistence level (in 2018–1.87 times) is evidence that the statutory subsistence level for citizens of Ukraine does not reflect the necessary actual expenditures of the population to meet basic needs.

The gradual increase of the subsistence level by the Government of Ukraine does not cover the expenses of the population to ensure normal functioning against the background of rapid outpacing rates of price growth.

Corteva Agriscience ^™^, the DowDuPont Agribusiness Unit and the The Economist Intelligence Unit (EIU) have published the results of the 2019 Global Food Security Index [63].

The issue of food security for Ukraine is now one of those that needs to be addressed in the near future.

Ukraine took 76rd place (GFSI total– 57.1) in 2019. At the same time, starting from 2013, the rating of Ukraine is constantly decreasing. Ukraine occupies the last place (26th) in the ranking of European countries in terms of GFSI [63, 73–80].

To analyze the economic affordability of food, the authors studied the trends in food security in Ukraine as a whole and the indicator of economic affordability as a component of the global food security index. This approach allows, according to the authors, a deeper understanding of the existing problems in the country.

The dynamics of the Global Food Security Index of Ukraine is shown in Fig 1.

**Fig 1:** Dynamics of the Global Food Security Index of Ukraine. Source: [63, 73–80]. Overall rank (0–113 where 1– most favourable); Score—weighted total of all category scores (0–100 where 100 –most favourable).

The Global Food Security Index characterises a country’s food security through four categories of indicators: affordability, availability, quality & safety, and natural resources & resilience. For the 2012–2019 period, Ukraine’s place in the global food security index has dramatically deteriorated by 32 positions in the ranking of the countries under study—from 44th place in 2012 to 76th in 2019. This happened despite the fact that the total score for all categories decreased by 2.3 over this period. During the 2017–2019 period, this indicator showed an increase of 2.0 points.

Positive changes in food security are occurring at a faster pace in other countries, meanwhile Ukraine’s social and economic policies are not conducive to improving the living standards of the population and achieving food security. The analysis of the components of the GFSI indicator of Ukraine in 2019 is characterised as follows: The best position of Ukraine is in the category of "quality & safety" (60th). Meanwhile, the categories of "availability" and "affordability" show a loss of position. In 2019, Ukraine occupied 89th and 71st positions in these indicators respectively (Fig 2).

**Fig 2:** Dynamics of the categories of the indicator of the Global Food Security Index of Ukraine. Source: based on [63, 73–80].

Since 2017, the GFSI has included the category of “natural resources & resilience”, according to which Ukraine ranked 77th place out of 113 countries in 2019. From the standpoint of social stability and the achievement of the country’s economic security, the category of "affordability" is important. Economic affordability of food demonstrates the economic ability to eat at a level that provides the necessary nutrients and energy from food.

During the study period, in the Ukraine’s food component of the Global Food Index—the category of "affordability" showed a decrease of 18 points.

The affordability of food includes a number of indicators: food consumption as a share of household expenditure, proportion of population under the global poverty line, gross domestic product per capita (USD PPP), agricultural import tariffs, presence of food safety net programs, and access to financing for farmers.

A study of food affordability as a component of food security will help to identify the risks and opportunities for achieving a higher level of food security. Let us focus on the characteristics of indicators that fall into the category of affordability and characterise the affordability of food for the population of Ukraine. Food consumption is a share of household expenditure. A study of the share of household expenditures on food purchases in total expenditures shows a gradual reduction. In 2020, it was 48.5% (Table 3).

**Table 3:** Calculation of indicators of the "affordability" category of GFSI.

Indicators	2000	2005	2010	2015	2016	2017	2018	2019	2020
GDP, bln. UAH	170.1	441.5	1082.6	1988.5	2383.2	2983.9	3558.7	3974.6	4194.1
Average annual official exchange rate of the hryvnia to the US dollar	5.4402	5.1247	7.9356	21.8447	25.5513	26.5966	27.2005	25.8456	26.957
GDP per capita, UAH	3436	9372	23600	46413	55848	70233	84190	94589,8	100432,5
Growth rates compared to the previous year,%	х	128.9	119.0	125.8	120.3	125.8	119.9	112,3	106.2
GDP per capita, USD	631.6	1828.8	2973.9	2124.7	2185.7	2640.7	3095.2	3659,8	3725,6
Growth rates compared to the previous year,%	х	128.9	119.0	125.8	120.3	125.8	117.2	118,2	101,8
Expenses / incomes per household per year, UAH	5012.4	14752.8	33277.2	59424.0	68644.8	82839.6	89257.2	106610.6	140047.1
Average household size, persons	2.76	2.61	2.59	2.58	2.58	2.58	2.58	2.58	2.58
Costs / incomes per person per year, UAH	1816.1	5652.4	12848.3	23032.6	26606.5	32108.4	34595.8	45993.0	47194.8
Growth rates compared to the previous year,%	х	136.6	115.3	122.3	115.5	120.7	107.7	132.9	102.6
Expenses / incomes per person per year, USD	333.8	1103.0	1619.1	1054.4	1041.3	1207.2	1271.9	1179.5	1750.7
Growth rates compared to the previous year,%	х	330.4	146.8	66.6	98.8	115.9	105.4	92.7	148.4
Food costs,%	64.0	56.6	53.5	57.9	54.3	53.1	50.9	49.1	48.5
Food costs per person per year, UAH	1162.3	3199.3	6873.9	13335.9	14447.3	17049.5	17609.3	17826.6	18291.9
Growth rates compared to the previous year,%	х	134.5	115.5	124.0	108.3	118.0	103.3	101.2	102.6
Food costs per person per year, USD USA	213.6	624.3	866.2	610.5	565.4	641.0	647.4	689.7	678.6
Growth rates compared to the previous year,%	х	292.2	138.8	67.5	92.6	113.4	101.0	106.5	98.3

Source: calculated by the authors [56–61, 81].

However, this level of food costs is much higher than the indicators of economically developed countries. Food Expenditures show significant differences in the structure of total household expenditures by decile (10%) groups depending on the size of the average per capita equivalent total income. Thus, for the first decile group (the lowest level of income), food costs account for 53.4% in the structure of total expenditures, but for the tenth group (high level of income), this indicator is at 33.9%. Thus, even for the tenth decile group, this indicator in Ukraine is almost three times higher than the average in EU countries.

A study of the structure of household cash expenditures suggests that in recent years there has been a redistribution of food expenditures, but the share of such expenditures remains high. At the same time, there is an increase in utility costs by more than 5% for the period under study. There are no changes in the costs associated with non-food goods and services, which are at the level of 32–33% of monetary expenditures. At the same time, the indicators of investment in construction, purchase of shares, etc. remain stable low during the study period—about 5% of total costs. Thus, we can conclude that the reduction of food costs is not as a result of approaching the optimal consumption of food and ensuring a balanced diet, but as a forced action caused by the need to cover other types of costs.

The EU-28 average [82] on the share of food expenditures over the last two decades is in the range of 12.0%–12.5% of the level of total consumer expenditures. In 2016, households in Luxembourg, Austria and Ireland spent the least on food in EU consumer spending—less than 10%. Lithuania, Estonia, and Bulgaria spent the most (about 20%).

For example, according to the Federal Statistical Office of Germany (Statistisches Bundesamt), the cost of food and tobacco products in 2020 averaged 15% of consumer spending.

Similar trends are typical for per capita expenditures/revenues per year. The total costs of the average Ukrainian in 2020 amounted to 47194.8 UAH or 1750.7 USD, which is 86.0% of the level of 2013 (2036.5 USD). On average, in 2020, one person in Ukraine spent $ 678.6 on food ($ 1.86 per day), which is 78.3% of the level of 2010. In the current conditions, it is impossible to ensure the affordability of food for the population of Ukraine.

Calculations have shown that food expenditures show a direct linear relationship with the level of GDP per capita:

Y=0.2252x+1016.8, (1)

The reliability of the obtained equation is confirmed by the value of the reliability of the approximation R^2^ = 0.9723.

The analysis between the level of income and food expenditure of the population of different decile groups is characterized by a linear relationship, which is described by the following equation:

Y=0.3257x+1469.5, (2)

The reliability of the obtained equation is confirmed by the value of the reliability of the approximation R^2^ = 0.9749. However, there are significant differences both in size and in share in the total cost of food in different decile groups depending on the size of the average per capita equivalent total income (Table 4).

**Table 4:** Total expenditure of households by decile (10%) groups depending on size of per capita equivalent total income, 2020 (on average per month per household, UAH).

Indicators	Decile (10%) groups									
	first (lower)	second	third	fourth	fifth	sixth	seventh	eighth	ninth	tenth (higher)
Total costs	4907	5847	6823	7342	8450	8811	9891	10048	11526	15190
Food costs	2790	3234	3680	3827	4138	4356	4784	4780	5297	5717
The share of food costs in total costs	56.9	55.3	54.1	52.1	48.9	49.5	48.4	47.6	45.9	37.6

Source: calculated by the authors based on [55, 60, 61]

For the first decile group, the highest share of food expenditures in total household expenditures is 56.9%. For the tenth decile it is 37.6% (the lowest), and the difference in food expenditure between them is 2.05 times.

The indicator of economic affordability of products Indicator of economic affordability of products (the share of total expenditures on food, including meals outside the home, in the total expenditures of households) in 2020 amounted to 49.2%. The limiting criterion for this indicator is considered to be its 60% level.

“Current food environments are creating inequities, and sustainable healthy foods are generally more accessible for those of higher socioeconomic status” [83]. Some studies from Hungary also concluded that healthy food choice depends on the education level of people and also the financial situation [45, 84].

In 2020, the food cost differentiation indicator was 159.0%. This is evidence that in Ukraine there is a significant gap (almost 1.6 times) in the differentiation of the cost of food by social groups. This figure is calculated as the ratio between the cost of food for 20 percent of the highest-income households and the cost of food for 20 percent of the lowest-income households.

Despite the high share of food expenditures in the structure of household expenditures, the population of Ukraine consumes basic food products less than the approved norms. This is typical for all food groups except for potatoes, vegetables and cucurbits (melons, cucumbers, gourds etc.) which are consumed above the norm by 8.1 and 1.9 percent, respectively. The lowest coefficients of satisfaction of demand are for fish and fish products and milk and dairy products– 0.620 and 0.531, respectively. Thus, the provision of daily energy needs is due to the consumption of cheap but high-calorie foods.

By 2013, inclusive, consumption of the basic food groups was gradually increasing. Deterioration in the volume and structure of consumption of the population of Ukraine began to occur starting from 2014. The year 2020 is characterised by a slight increase in the consumption of meat and meat products, milk and milk products, oil. Dynamics of consumption, rational norm of consumption (RNC) and satisfaction coefficient of needs (SCN) for separate products are given in Table 5.

**Table 5:** Dynamics of food consumption by the population of Ukraine (per capita per year; kilograms).

Main food-stuffs	RNC	Years									SCN
		2000	2005	2010	2015	2016	2017	2018	2019	2020	
Meat and meat products	83	32.8	39.1	52.0	50.9	51.4	51.7	52.8	53.6	53.8	0.648
Milk and milk products	380	199.1	225.6	206.4	209.9	209.5	200.0	197.7	200.5	201.9	0.531
Eggs, pcs	290	166	238	290	280	267	273	275	282	278	0.959
Fish and fish products	20	8.4	14.4	14.5	8.6	9.6	10.8	11,8	12.5	12.4	0,620
Sugar	38	36.8	38.1	37.1	35.7	33.3	30.4	29.8	28.8	27.8	0.732
Oil	13	9.4	13.5	14.8	12.3	11.7	11.7	11.9	12.0	12.3	0.946
Potatoes	124	135.4	135.6	128.9	137.5	139.8	143.4	139.4	135.7	134.0	1.081
Vegetables and cucurbits crops	161	101.7	120.2	143.5	160.8	163.7	159.7	163.9	164.7	164	1.019
Fruits, berries and grapes (without processed for wine)	90	29.3	37.1	48.0	50.9	49.7	52.8	57,8	58.7	56.5	0.628
Bread-stuff products (bread and macaroni counted as flour; cereals, flour, legumes)	101	124.9	123.5	111.3	103.2	101.0	100.8	99.5	97.6	96.6	0.956

Source: calculated by the authors based on [54, 56–60].

A comparison of the data in Tables 5 and 6 shows the possibility of increasing food consumption to ensure a balanced diet of the population of Ukraine. The actual data show that at the maximum value of the daily caloric content of food products of animal origin 1375 calories for the population of Ukraine, this figure is within 790 calories (1.7 times lower). At the maximum value of the daily caloric content of products of plant origin—1125 calories, the daily caloric content of vegetable products of the average Ukrainian—1952 calories (1.7 times higher). The caloric content of products of animal origin does not exceed 30% of the actual daily caloric content of the diet of the average Ukrainian at a rate of 55%. Thus, we can conclude that changes in the structure of consumption and deviations of consumption of certain products from rational norms are caused by low incomes, rather than food preferences.

**Table 6:** Food consumption by the population of Ukraine, Russia and Belarus.

Basic products	Per capita per year; kilograms		
	Ukraine	Russia	Belarus
Meat and meat products	53.6	91	97
Milk and milk products	201.9	267	246
Eggs, pcs	278	234	264
Vegetables, water-melons and gourds	164.7	104	152
Fruits, berries and grapes	58.7	76	97
Potatoes	134.0	58	175

Source: calculated by the authors based on [55, 85, 86]

Comparisons of the consumption of basic food products by the population of Ukraine, Belarus and Russia in 2019 are presented in Table 6.

Apparently, the population of Ukraine has the lowest level of consumption of meat and meat products, milk and dairy products. Meat and meat products in Ukraine are consumed 45% less than in Belarus and 41% less than in Russia. Milk and dairy products are most consumed by the population of Russia, which is 24% higher than in Ukraine. The most balanced is the nutrition of the population of Belarus.

A lower level of food consumption per capita in Ukraine is observed even despite the fact that food expenditures in Ukraine were the highest in 2019–49.1% of total household expenditures. In 2019, according to official statistics, food expenditures by households in Russia amounted to 34.6%, and in Belarus—35.7% of total household expenditures. The given indicators testify to the discrepancy between food prices and the level of income of the population of Ukraine.

Performance of countries based on their 2019 food security score are Belarus—36th and Russia—42nd places in GFSI rank. These countries have affordability rates of 76.0 and 79.8, respectively. Instead, Ukraine ranked 76th in the GFSI rank and had an affordability score of 63.9 (maximum 100).

The main tasks in increasing the economic affordability of food for the population of Belarus are:

- further reduction of public spending on food;
- threats to food affordability in the face of growing urbanization [21, p. 15];
- significant share of food imports—21% [87, p.38].
- For Russia, the main problems of ensuring the affordability of food are:
- low level of self-sufficiency of the country with food;
- a number of unresolved issues at the state level;
- territorial imbalance in the location of production of raw materials and processing facilities [88, p.185];
- significant differences in regional income levels, which determines the level of household spending on food. If on average in Russia 21% of families spend more than 50% of all consumer spending on food, in some republics this figure is 3–4 times higher (83.9% of families in Ingushetia, the Chechen Republic—64%, Dagestan—60%);
- a significant decrease in food imports due to the introduction of sanctions;
- lack of investment funds to ensure an effective food import substitution policy [89, p.118].

The results show that the prevailing trends in household food consumption are determined by the level of their affordability. For Ukrainian households, food consumption depends on both income levels and prices. Food products are essential goods, the consumption of which should be insensitive to income, so the volume of demand should not respond to changes in income.

Consumption of bread, bakery products and sugar will decrease from the surveyed goods with the growth of the income level. Such behavior is typical for goods of lower consumer value. Thus, with an increase in the level of income, these products will be replaced in the diet.

All other foods show a high dependence of consumption on income. This situation is typical for normal products to which food products do not belong.

In most of the developed countries of the world, the demand for the main groups of food products is inelastic not only in terms of price, but also in terms of income. With an increase in per capita income, the demand for this group of goods grows, but not in direct proportion to the increase in income. Other expenditures are growing at a significantly higher rate: for clothing, durable goods, services, savings, and the like.

At the same time, the main reason for the decrease in the consumption of food products by the population was the low level of purchasing power, which is confirmed by the calculations presented in Table 3, since the level of self-sufficiency of Ukraine in the basic types of food (produced for domestic use) in recent years has exceeded 100%, with the exception of fruits, berries and grapes;milk and milk products. Self-sufficiency level is shown in Table 7.

**Table 7:** Self-sufficiency by basic food-stuffs in 2020 (output for domestic use).

Basic products	Self-sufficiency rate,%		
	Ukraine	Russia	Belarus
Meat and meat products	110.1	98	133
Milk and milk products	99.1	84	241
Eggs	125.0	97	128
Vegetables, water-melons and gourds	104.6	90	107
Fruits, berries and grapes	75.9	39.4	48
Potatoes	100.1	102	111
Grain	323.3	99.1	85,4

Source: calculated by the authors based on [7, 55, 61, 90];

Comparative analysis makes it possible to conclude that Russia has the lowest indicators of self-sufficiency in basic food products in comparison with Ukraine and Belarus. Although Ukraine demonstrates a sufficient level of self-sufficiency in basic food products, it has a lower level of self-sufficiency in most products than Belarus, with the exception of grain and fruits, berries and grapes.

The current level of self-sufficiency in basic foodstuffs is an important prerequisite for ensuring economic security and affordability of food. The low level of purchasing power of the population forms an excess supply of food products in the domestic market of Ukraine. Under these conditions, food producers can focus on the following actions:

1. reduction of excess supply in the domestic market to maintain the existing price level;
2. reduction of prices for ready-made food products to stimulate demand, for those food products that are consumed at a level lower than rational consumption rates;
3. expansion of export opportunities for the sale of manufactured products outside Ukraine.

Each of the possible behaviors of food producers can have different effects on the economic affordability of food. Most food producers are trying to keep the current level or increase production by expanding export opportunities. This strategy leads to an increase in domestic prices and, consequently, limits the purchase of domestic producers (this is typical for poultry, oil, eggs).

Reduction of supply does not ensure the stability of demand, there is a replacement of imported products (dairy products).

Reducing prices to stimulate demand for bread and bakery products allows companies to make a profit due to the scale of production.

In turn, the gradual increase in income will stimulate domestic demand and shape the affordability of food. A high level of income will ensure a balanced diet.

To determine the impact of income levels on the consumption of certain foods, the authors analysed the time series for the period 2000–2020 and determined the correlation dependence between the level of income and consumption of certain food products. The results obtained indicate the following: the greatest dependence on the level of income was shown by the consumption of fruits, berries, grapes; meat and meat products; vegetables and cucurbits; and eggs. For these groups of goods, increasing income levels will increase consumption. These goods have a high level of income elasticity and they belong to the category of normal.

Consumption of oil and other vegetable fats, fish and fish products (neutral products) does not depend on the level of income. But the consumption of bread and bakery products; sugar, milk and dairy products will decline with increasing income levels. The decrease in the consumption of bread and bakery products and sugar can be explained by the fact that these products are classified as goods for which demand is inversely proportional to consumer income. Milk and dairy products will be replaced by increased consumption of meat and meat products.

To determine the relationship between the level of income and consumption of certain foods, where a dense correlation was found, a regression equation was constructed and the type of relationship was determined (Fig 3).

**Fig 3:** The equation of the relationship between the consumption of certain foods and the income level of the population. Source: calculated by the authors.

A considerable proportion of the population is under the global poverty line. According to official statistics, 29.5% of households were below the actual subsistence level in 2020. At the same time, the percentage of households with per capita equivalent total monthly income lower than the actual subsistence level living in rural areas was 3.0% higher than in those living in cities. In addition, the actual subsistence level in 2020 was 70.8% of the average level of per capita equivalent total household income (Table 8).

**Table 8:** Distribution of households by per capita equivalent total income (on average per month).

	All households				including those living							
					in cities				in rural areas			
	2017	2018	2019	2020	2017	2018	2019	2020	2017	2018	2019	2020
Average level of per capita equivalent total income, UAH	3797.7	4606.8	5743,4	5920.1	3880.4	4772.2	6053,9	6186,4	3637.5	4283.5	5132.3	5369.2

Source: calculated by the authors based on [52–55].

Rapid growth rates of prices are not conducive to increasing the affordability of food products.

Thus, relative to the 2010 level, the increase in food prices was more than 2.2 times (Fig 4). And although income per capita grew at a high rate (2.7 times over this period), this did not cause significant changes in the consumption of basic food products.

**Fig 4:** Price indices, % by 2010. Source: developed by the authors according to [54, 56–60].

Economic affordability of food is also characterised by the gross domestic product per capita indicator (USD PPP). According to the above statistics, GDP per capita in Ukraine in UAH is growing at a fairly high rate, however, taking into account the average annual official exchange rate of the hryvnia against the USD, the change in this indicator has the following form: by 2013 this indicator grew from 631.6 in 2000 up to 4187.8 USD, but starting from 2014, GDP per capita in USD shows a decline and, in 2018 it amounted to 2640.7 USD– 63.1% against the indicator of 2013. This trend is associated with the military actions in the East of Ukraine; negative processes in the economy; the deployment of inflationary processes, and the devaluation of the hryvnia.

Thus, the considered indicators that determine the economic affordability of food indicate the existence of food insecurity at the level of individual households, characterised by low incomes and, consequently, limited access to food.

Today, the nutrition of the population of Ukraine is characterized by an unsatisfactory structure, as the ratio between the consumption of macro- and micronutrients, namely the ratio between proteins, fats and carbohydrates, which should be within: 1: 1.2: 4.6. Actual data indicate a ratio of 1: 1.6: 4.4. Thus, fat intake is lower with increased carbohydrate intake. In addition, the proportion of animal proteins should be at least 50% of the total amount of protein consumed, and the ratio between animal and vegetable fats should be 75%–25%. These requirements for a balanced diet are also violated in Ukrainian households and amount to 30:70.

## 5. Conclusions

The lack of adequate financial assets (household income) that could compensate for the decrease in income leads to an increase in the economic danger of households. This is exactly the situation in most households in Ukraine. The state of economic security is influenced by factors that are in constant motion and determine the state’s ability to protect the interests of the population, the key subjects of economic relations. Economic security is the basis of the national security of the state. The prevention and overcoming of economic danger should be one of the priority tasks of the state social policy.

The low level of food security in Ukraine is formed by interrelated factors. It is determined by the low level of GDP per capita; low incomes of the population; the high share of food expenditures in the structure of population expenditures fails to provide economic affordability of food for the population; and also the lack of an effective program to ensure food security at the country level.

Various indicators are used in scientific publications to characterise the state of economic security, one of which is the indicator of economic danger (instability). Economic instability refers to the uncertainty associated with people’s lives. Limited economic affordability of consumption affects the state of economic danger. Overcoming economic instability and minimising the possible consequences of economic instability is one of the main tasks of economic security.
